This article has been retracted.

# Camrelizumab and Apatinib Combined with Radiotherapy Is Effective in Advanced Oligometastatic Non-Small-Cell Lung Cancer

**DOI:** 10.1155/2022/5067402

**Published:** 2022-09-24

**Authors:** Wei Ye, Zhonghua Song, Zhongkun Lin

**Affiliations:** ^1^Respiratory Medicine, Shandong Provincial Third Hospital, Jinan 250031, Shandong, China; ^2^Department of General Practice, Shandong Provincial Third Hospital, Jinan 250031, Shandong, China; ^3^Department of Oncology, Shandong Provincial Third Hospital, Jinan 250031, Shandong, China

## Abstract

**Objective:**

To investigate the effect of camrelizumab + apatinib combined with radiotherapy on the expression of TRIM27, SCC-Ag, and CYFRA21-1 in advanced oligometastatic non-small-cell lung cancer (NSCLC).

**Methods:**

A retrospective analysis of patients with oligometastatic NSCLC who were treated at our hospital from January 1, 2021, to March 31, 2022. Patients who met the inclusion criteria were summarized into an observation group (camrelizumab on the basis of the control group), or a control group (radiotherapy combined with oral apatinib). The disease control rate, immune function, changes in the levels of TRIM27, SCC-Ag, CYFRA21-1, and the occurrence of adverse effects were compared between the two groups.

**Result:**

There were 86 patients who met the inclusion criteria, with 53 cases in the observation group and 33 cases in the control group. There were significant differences in complete remission (CR, 25/53 vs. 10/33), partial remission (PR, 17/53 vs. 12/33), disease control (DC, 7/53 vs. 4/33), disease progression (DP, 4/53 vs. 7/33), and disease control rate (49/53 vs. 26/33) between the observation group and the control group. There was no significant difference in immune function between the two groups before treatment (*p* > 0.05). After treatment, the levels of CD3^+^, CD4^+^, CD4^+^/CD8^+^*t* cells, and NK cells in the observation group were higher (*p*=0.015, 0.035, 0.003, 0.001, respectively), while the level of CD8^+^*t* cells was lower (*p* < 0.001). There were no significant differences in TRIM27, SCC-Ag, or CYFRA21-1 between the two groups before treatment (*p* > 0.05). After treatment, the observation group had lower levels of TRIM27 (*p*=0.035), SCC-Ag (*p*=0.045), and CYFRA21-1 (*p*=0.003). There was no significant difference in the occurrence of adverse events between the two groups (*p* < 0.05).

**Conclusion:**

Treatment of camrelizumab + apatinib combined with radiotherapy is effective for advanced oligometastatic NSCLC, with mild adverse effects.

## 1. Introduction

Non-small-cell lung cancer (NSCLC) is a malignant tumor with high mortality, accounting for about 85% of all lung cancer patients in the United States and Europe. Most patients have distant metastases at the time of diagnosis, thus losing the window of complete cure [1–4]. The idea of oligometastases was first proposed in 1995 [5], which believed that cancer in this stage was only limited to one or a few targeted metastases. At present, there is no standard for the definition of oligometastases, but the European Society of Oncology and some recent studies believe that as long as the location of the metastases and the number of metastatic tissues (< 5), oligometastases can be confirmed by a complete radiological examination [6, 7]. Oligometastasis is a transitional period in which the local primary tumor spreads to a larger area, and it has the potential to be cured. Squamous cell carcinoma antigen (SCC-Ag) is a tumor-related antibody produced when tumor cells are abnormally differentiated, and it can accelerate the proliferation of their DNA. Cytokeratin 19 fragment antigen 21-1 (CYFRA21-1) is a major cytoskeletal protein, which can accelerate the adhesion of cancer cells by inhibiting apoptosis and increasing its content and pass [8]. This study retrospectively analyzed the oligometastatic NSCLC patients treated at our hospital.

## 2. Materials and Methods

### 2.1. General Information

A retrospective analysis of patients with oligometastatic NSCLC who were treated in our hospital from January 1, 2021, to March 31, 2022. This study was approved by the Institutional Ethical Committee of Shandong Provincial Third Hospital. All patients in this study signed the informed consent forms. The inclusion criteria were as follows: (1) pathologically confirmed stage VI NSCLC; (2) signed informed consents; and (3) with complete data. The exclusion criteria were as follows: (1) patients with mental disorders; or (2) severe organ failure; or (3) lost to follow-up.

Patients in the control group were given radiotherapy combined with oral apatinib (Jiangsu Hengrui Medicine Co., Ltd., approved by H20140103), with an initial dose of 250 mg/d. If no adverse effects, it will be increased to 500 mg/d, 28 days as a cycle, and the treatment will be continued for 4 cycles. Patients in the observation group were treated with camrelizumab (Suzhou Shengdia Biopharmaceutical Co., Ltd., S20190027) on the basis of the observation group, given by iv., 200 mg each time, once every 3 weeks, for continuous treatment of 4 cycles.

1. After 4 cycles of treatment, the curative effect of patients was evaluated according to the World Health Organization tumor curative effect evaluation standard [9]. Complete remission (CR): complete disappearance of all target lesions in the patient. Partial remission (PR): the longest diameter of the target lesion was reduced by 20% to 30% compared with the time of admission. Disease progression (DP): the longest diameter of the target lesion increased by 20% to 30% compared with admission. Disease Control (DC): between CR and DP. Disease control rate is the sum of CR rate, PR rate, and DC rate;
2. Before treatment and after 4 cycles of treatment, an American FACS-type flow cytometer was used to detect immune function indicators, including CD3^+^, CD4^+^, CD8^+^, CD4^+^/CD8^+^, and natural killer (NK) cell levels;
3. Enzyme-linked immunosorbent assay (ELISA) was used to detect serum SCC-Ag and CYFRA21-1 levels; TRIM27 was detected by the RT-PCR method [10].
4. Record the occurrence of adverse effects during the treatment, including gastrointestinal discomfort, abnormal liver and kidney function, leukopenia, and thrombocytopenia.

### 2.2. Statistical Methods

The data in this experiment need to be verified by SPSS21.0 (SPSS, Chicago, IL, USA) software. The data by count were tested by the *χ*^2^ test, and the data by measurement were tested by *t*-test. *p* < 0.05 (2-tailed) was used as the threshold for statistical significance.

## 3. Results

### 3.1. General Information

In total, 489 patients with stage IV NSCLC were treated in our hospital from January 1, 2021, to March 31, 2022, including 86 patients with oligometastatic NSCLC who met the inclusion criteria and were summarized into 2 groups according to the treatment method. The observation group (53 cases, including 29 males and 24 females, aged 43.05 ± 1.39 years) and the control group (33 cases, including 18 males and 15 females, aged 42.87 ± 1.92 years). There were no significant differences in gender, age, and BMI between the two groups (*p* > 0.05, Table 1).

### 3.2. Comparison of Disease Control Rates between the Two Groups

There were significant differences in CR (25/53 vs. 10/33), PR (17/53 vs. 12/33), DC (7/53 vs. 4/33), DP (4/53 vs. 7/33), and disease control rate (49/53 vs. 26/33) between the observation group and the control group (*p* < 0.001). See Table 2 for details.

### 3.3. Comparison of Immune Function between the Two Groups

There was no significant difference in immune function between the two groups before treatment (*p* > 0.05). After treatment, there were significantly higher CD3^+^*t* cells (59.29 ± 3.31 vs. 51.89 ± 2.41), CD4^+^*t* cells (32.79 ± 2.81 vs. 25.23 ± 2.66), CD4^+^/CD8^+^*t* cell (1.41 ± 0.59 vs. 1.14 ± 0.52), and NK cells (18.26 ± 3.51 vs. 14.26 ± 3.14) and lower CD8^+^*t* cell (23.63 ± 1.31 vs. 23.97 ± 1.36) in the observation group. See Table 3 for details.

### 3.4. Comparison of the Levels of TRIM27, SCC-Ag, and CYFRA21-1 between the Two Groups

There was no significant difference in the index levels between the two groups before treatment (*p* > 0.05). After treatment, there were lower TRIM27 (0.35 ± 0.03 vs. 0.51 ± 0.04), SCC-Ag (1.29 ± 0.34 vs. 1.51 ± 0.36), CYFRA21-1 (1.93 ± 0.31 vs. 2.39 ± 0.47) (*p*=0.035, 0.045, and 0.003, respectively). See Table 4.

### 3.5. Comparison of Adverse Effects between the Two Groups

There was no significant difference in the occurrence of adverse effects between the two groups (*p* < 0.05). See Table 5.

## 4. Discussion

In the early stage of NSCLC, there may be no obvious clinical signs for early diagnosis. With the latent development of the disease, most patients will have abnormalities in CT or chest X-ray examinations. However, they are in the late stage of cancer, missing the opportunity for treatment and radiation therapy, and the 5-year survival rate is only 20% [11–14]. The occurrence of NSCLC is the main cause of local pain, compression symptoms, and mass effect, which increases the tumor burden and greatly reduces the quality of life. However, in patients with oligometastatic NSCLC, due to the transition period from primary metastasis to large-scale metastasis, the metastatic site and metastatic tissue structure are relatively simple, and the tumor burden is relatively light during this period. In combined therapy, there is good tolerance and a good prognosis.

The pathogenesis of NSCLC is still unclear, but the abnormal expression of tumor proteins related to NSCLC may cause abnormal proliferation of epithelial cells, thereby causing changes in their transcription. SCC-Ag is a glycoprotein secreted in dividing tumors, and its expression may be increased during rapid proliferation or marked differentiation. CYFRA21-1 is an active substance with enhanced tumor cell morphology, and its role is to enhance tumor cell infiltration into the basement membrane and epithelial-mesenchymal transition [15]. TRIM27 can activate the NF-*κ*B signaling pathway and activate the transcription of the downstream target genes DKK1 and c-Myc of the Wnt/*β*-catenin pathway, thereby promoting their proliferation and activation. TRIM27 can also promote the proliferation of NSCLC, thereby activating the expression of ERK and JNK signal transduction pathways, thereby enhancing the infiltration of NSCLC [16–18].

The apatinib used in this study, as a new drug with its own patent, was first approved as third-line chemotherapy in November 2014. Clinical trials have shown that it has a significant efficiency. In addition, apatinib is an oral tyrosine kinase inhibitor (TKI), which has the advantages of simple use, small side effects, safety, and reliability. Due to more and more relevant clinical trials, apatinib is gradually being applied to the clinical treatment of advanced NSCLC. Camrelizumab is a new type of NSCLC drug newly developed in China. It can be combined with PD-1 to inhibit its interaction with apoptosis receptors and improve the body's immunity [19, 20]. In patients with NSCLC, the long-term use of drugs and the weakening of the immune system will cause the decline of the immune system, thereby aggravating the general condition of NSCLC [21]. Therefore, it is very necessary to strengthen immunotherapy for non-small-cell lung cancer. Retrospective analysis of the combined treatment methods adopted by the observation group in this study achieved excellent clinical effects, effectively reduced the levels of TRIM27, SCC-Ag, and CYFRA21-1, and improved the immune function of the subjects. At the same time, there was no significant difference in the statistics of adverse effects between the two groups. It might need further investigation for those therapies in complicated cases [22–27].

In general, camrelizumab + apatinib combined with radiotherapy for advanced oligometastatic non-small-cell lung cancer has good efficacy, mild adverse effects, high safety, and can be widely used.

## Figures and Tables

**Table 1:** General information of the two groups.

Group	Male/Female (example)	Average age (years)	BMI (kg/m^2^)
Observation group (*n* = 53)	29/24	43.05 ± 1.39	24.73 ± 3.44
Control group (*n* = 33)	18/15	42.87 ± 1.92	23.96 ± 3.32
*t*/*χ*^2^	8.257	10.371	4.374
*p*	0.391	0.853	0.389

**Table 2:** Comparison of disease control rates between the two groups (cases, %).

Group	CR	PR	DC	DP	Disease control rate
Observation group (*n* = 53)	25 (47.17)	17 (32.08)	7 (13.21)	4 (7.55)	92.45
Control group (*n* = 33)	10 (30.30)	12 (36.36)	4 (12.12)	7 (21.21)	78.79
*χ * ^2^	—	18.736			
*p*	—	<0.001			

**Table 3:** Comparison of immune function between the two groups ($\bar{x}$ ± *s*).

Group	Observation group (*n* = 53)		Control group (*n* = 33)		*t*	*p*
	Before therapy	After treatment	Before therapy	After treatment		
CD3^+^ (%)	56.36 ± 2.43	59.29 ± 3.31	56.39 ± 2.46	51.89 ± 2.41	10.649	0.015
CD4^+^ (%)	28.06 ± 2.75	32.79 ± 2.81	28.13 ± 2.72	25.23 ± 2.66	7.287	0.035
CD8^+^ (%)	26.83 ± 1.62	23.63 ± 1.31	26.78 ± 1.66	23.97 ± 1.36	9.468	0.003
CD4^+^/CD8^+^	1.23 ± 0.32	1.41 ± 0.59	1.25 ± 0.34	1.14 ± 0.52	9.521	0.001
NK cells (%)	16.47 ± 3.32	18.26 ± 3.51	16.39 ± 3.32	14.26 ± 3.14	13.739	<0.001

**Table 4:** Comparison of TRIM27, SCC-Ag, and CYFRA21-1 levels between two groups ($\bar{x}$ ± *s*).

Group	Observation group (*n* = 53)		Control group (*n* = 33)		*T*	*p*
	Before therapy	After treatment	Before therapy	After treatment		
TRIM27	0.83 ± 0.07	0.35 ± 0.03	0.82 ± 0.06	0.51 ± 0.04	16.798	0.035
SCC-Ag (*μ*g/L)	1.76 ± 0.46	1.29 ± 0.34	1.75 ± 0.42	1.51 ± 0.36	11.619	0.045
CYFRA21-1 (*μ*g/L)	3.95 ± 0.83	1.93 ± 0.31	3.97 ± 0.86	2.39 ± 0.47	8.549	0.003

**Table 5:** Comparison of adverse effects between the two groups (cases, %).

Group	Gastrointestinal discomfort	Abnormal liver and kidney function	Leukopenia	Thrombocytopenia
Observation group (*n* = 53)	10 (18.87)	9 (16.98)	7 (13.21)	11 (20.75)
Control group (*n* = 33)	6 (18.18)	5 (15.15)	5 (15.15)	7 (21.21)
*χ * ^2^	11.781	16.392	9.284	14.163
*p*	0.824	0.856	0.733	0.945

## Data Availability

The data can be obtained by direct contact with the corresponding author.
